# Effect of Continuous Care Combined with Constraint-Induced Movement Therapy Based on a Continuing Care Health Platform on MBI and FMA Scores of Acute Stroke Patients

**DOI:** 10.1155/2022/5299969

**Published:** 2022-01-25

**Authors:** Pan Yingying, Lixin Zang, Xiaojie Wang, Xiuqin Yang

**Affiliations:** ^1^Linyi Central Hospital, Linyi, Shandong Province 276400, China; ^2^Feicheng Hospital Affiliated to Shandong First Medical University, Feicheng, Shandong Province 271600, China; ^3^Respiratory Medicine, Qingdao Eighth People's Hospital, Qingdao, Shandong Province 271600, China; ^4^Qingdao Municipal Hospital, Qingdao, Shandong Province 266000, China

## Abstract

**Methods:**

68 acute stroke patients admitted to our hospital from July 2018 to July 2019 were selected as the study participants and divided into group A and group B based on the odd and even numbers of their admission numbers, with 34 cases in each group. Patients in group B accepted the routine rehabilitation exercise, while patients in group A accepted the continuous care combined with constraint-induced movement therapy (CIMT) under a health platform, so as to compare their upper limb function recovery by the Fugl–Meyer assessment (FMA) and improved median Barthel index (MBI).

**Results:**

The general information of the two groups were not obviously different (*P* > 0.05) but comparable; after intervention, the FMA scores (38.42 ± 7.62 vs 31.22 ± 7.25) and MBI scores (78.63 ± 6.52 vs 70.24 ± 6.48) of patients in group A were significantly higher than those of group B (*P* < 0.001); the activities of daily living (ADL) and trunk control test (TCT) scores at T1, T2, and T3 of group A were significantly higher than those of group B (*P* < 0.05); at 6 months after discharge, the self-concept, self-care skills, self-care, self-responsibility, health knowledge level, and total ability scores of patients in group A were significantly higher than those in group B (*P* < 0.05); the Generic Quality of Life Inventory-74 (GQOL-74) scores after intervention of the two groups were significantly higher than those before intervention (*P* < 0.05) and those of group A were significantly higher than those of group B (72.13 ± 4.69 vs 63.19 ± 4.72; *P* < 0.05); when comparing with group B, group A presented significantly higher walking speed and gait period and lower support phase (*P* < 0.05).

**Conclusion:**

The combination of continuous care and CIMT under a health platform can effectively promote the rehabilitation of upper limb functions and improve the activities of daily living and trunk control for acute stroke patients, with an effect better than conventional rehabilitation exercises, which is worthy of promotion.

## 1. Introduction

Acute stroke is a sudden cerebral ischemic disease with rapid progress, which refers to the cerebrovascular injury caused by multiple factors, and the prevention of recurrence and functional recovery are the focuses of daily care for acute stroke patients [1]. With the constant advances in the treatment of cerebrovascular diseases in recent years, the survival rate of stroke patients has improved significantly, but most survivors still have different degrees of nerve, limb, and social function disorders. The recovery of lower limb motor functions in acute stroke patients with hemiplegia tends to be better than that of the upper limbs, which is due to the fact that most upper limb movements are precise, leading to a slower recovery rate. Moreover, the exercises on the upper limbs are usually overlooked as patients pay more attention to the recovery of walking and lower limb function in the early stages, so upper limb disorders seriously affect patients' quality of life and become a major concern in the medical community [2, 3]. Rehabilitation treatment after discharge is required for most patients as this disease is difficult to cure. However, if their family members lack relevant knowledge about acute stroke nursing, better nursing cannot be provided, and patients cannot effectively manage their health behaviors out of hospital by themselves, thus seriously affecting the recovery. Continuous care, an extension of the inpatient care service, provides health guidance for discharged patients and promotes their recovery progress. In addition, constraint-induced movement therapy (CIMT) is effective in improving the motor function of patients with ipsilateral hemiplegia and promoting rehabilitation by stimulating the motor function of the affected hemiplegic limb and increasing the excitability and responsiveness of the nervous system [4]. A large number of clinical studies have confirmed that [5] combining multiple rehabilitation therapies is required to achieve the optimal treatment effect as a single rehabilitation therapy cannot exert the ideal efficacy. Therefore, this study aimed to investigate the effects of continuous nursing combined with CIMT by a health platform on the limb motor function and quality of life in acute stroke patients.

## 2. Materials and Methods

### 2.1. Clinical Characteristics

68 acute stroke patients admitted to our hospital from June 2018 to July 2019 were selected as the research objects and divided into group A and group B based on the odd and even numbers of their admission numbers, with 34 cases in each group. The clinical characteristics of patients in both groups are shown in Table 1.

### 2.2. Inclusion Criteria

The inclusion criteria were as follows: (1) patients who met the relevant diagnosis criteria in the rehabilitation treatment of stroke [6]; (2) patients who had the disease for the first time; and (3) patients who had stable vital signs and no progression of symptoms. The study was approved by the hospital ethics committee, and patients signed informed consent.

### 2.3. Exclusion Criteria

The exclusion criteria were as follows: (1) patients with a history of seizure or psychiatric disorder; (2) patients with kidney, liver, or other organ failure; (3) patients with poor compliance or cooperation; and (4) patients with consciousness or cognitive impairment.

### 2.4. Intervention

#### 2.4.1. Control Group

According to the operation specification for common rehabilitation technology [7], conventional rehabilitation exercises were given to patients in group B, including stand training, kneeling training, lying position training, and balance training. The subjective exercise intensity was measured by the *Rating of Perceived Exertion* [8] (RPE scale), which was appropriate at levels 11–13. The 60-minute exercise (with each training lasting 15 min) was carried out once a day for 6 months. The patients were followed up by telephone every two weeks to understand the rehabilitation situation.

### 2.5. Intervention Group

Patients in the intervention group were given continuous care combined with CIMT under a health platform for 6 months. The nurses taught the patients how to use the mobile health platform when patients are in hospital.

### 2.6. Construction of Mobile Health Platform Team

The mobile health platform team consisted of the project leader and 2 postgraduate students and was constructed with 4 modules, namely, a self-management feedback module, a nurse-patient communication support module, a health information transmission module, and an outpatient follow-up assistant. After the initial construction of the platform, 2 chief physicians with more than 6 years of medical experience, 3 chief physicians, and 5 senior nurses objectively evaluated the setup and operation modes of the platform and gave relevant modification opinions. When the problems were modified, patients could access and use the platform and were interviewed after using it for one week to obtain the following information in the form of a semistructured investigation: (1) whether the platform structure setup was reasonable and was there any inconvenience during use; (2) after using the platform, did patients obtain any practical progress in self-monitoring, disease knowledge, self-symptom management, etc.; (3) were there any advises on the improvement of subsequent maintenance of the platform; and (4) reasons for less frequent use. The mobile health platform was completed and modified by summarizing the interview results and maintained and managed by 2 clinical nurses.

### 2.7. Content and Use of the Mobile Health Platform

Patients followed the official account of the acute stroke health platform to enter the database and recorded their basic clinical information including name, bed number, age, and admission time. (1) Health information transmission included push messages of acute stroke knowledge base, recovered cases tracking, and weekly popularization of disease knowledge. The push contents were edited by clinical nurses and published after being reviewed by the attending doctor of the department, and should be universal, scientific, and straightforward for patients and their family members. The acute stroke knowledge base should include overview, causes, clinical treatment principles, self-monitoring methods, motor rehabilitation, and follow-up management of acute stroke. The weekly popularization of disease knowledge was mainly delivering the latest news of acute stroke treatment to patients, such as the latest diagnosis and treatment guidelines for acute stroke at home and abroad, and with the help of the analysis of acute stroke caused by different factors and the summary of assisting diagnosis and treatment, prognosis after discharge, self-management situation, and by the recovered case tracking function, patients would form an intuitive understanding of the self-management behaviors and diagnosis and treatment of the disease. The abovementioned health information could be found by clicking the “Heart Protection Helper” and then directly clicking the title. (2) The self-management feedback module urged patients to upload their self-checking results, including blood pressure, heart rate, body weight, and sleep quality. And clinical nurses reviewed the information and dealt with the abnormal signs in time. (3) The nurse-patient communication support module received consultation via message or e-mail from patients and their family members. Clinical nurses checked the messages or e-mails of the health platform at least 3 times a week, so as to inform patients about the importance of timing and quantitative drug use and notify the attending doctors to change the drugs or adjust the dosage. (4) With the outpatient follow-up assistant, patients' drug plans were optimized and adjusted according to the latest rehabilitation treatment of stroke [9], and a message would be sent to patients automatically 2 weeks after discharge to remind them to go to the stroke-specific clinic, with the specific process and address attached.

During CIMT, patients wore a home-made sling or glove on the healthy side that restricted the movement of their wrist and upper limb for more than 90% of their waking time every day, and took them off only when bathing, going to the toilet, sleeping, etc. The rehabilitation nursing staff assisted the patients to change their body position and placement of good limbs regularly, helped to suspend the healthy leg, and instructed the patients to carry out the following exercises: plate exercise involving stepping and hip lifting with the affected foot for 5–10 min each time and once a day; slow passive movement of upper and lower limbs step by step for 10 min each time and twice a day; walking exercise in a standing position for 15 min each time and twice a day; and balance exercise in a sitting position for 15 min each time and twice a day. Finally, 1–2 shaping movements were selected to make a specific rehabilitation scheme according to patients' clinical conditions, including 5–10 min of stretching and relaxing exercise before training. The rehabilitation exercises were done 5 consecutive days a week for 6 months.

### 2.8. Observation Indexes

The upper limb functions of patients in both groups were evaluated by the Fugl–Meyer assessment (FMA) scale [10] and the median Barthel index (MBI) [11], of which the items in the FMA scale (0–66 points) included upper limb, flection, pronation, and shoulder abduction, and the 12 items of the MBI (0–100 points) included showering, getting dressed, and personal hygiene, with higher scores indicating better recovery of patients' upper limb function.

The activities of daily living of patients in both groups were evaluated before intervention (T0), 1 month after intervention (T1), 3 months after intervention (T2), and 6 months after intervention (T3) by the activity of daily living (ADL) scale [12] (0–100 points), which included 10 items such as eating, getting dressed, and defecation control, with higher scores indicating better ADL.

The trunk control of patients at different times was evaluated by the trunk control test (TCT) [13], in which there were 4 steps and each step was divided into 3 grades, with 0 point indicating the patient was unable to perform movement without assistance, 12 points indicating the patient was able to perform movement with a little help (for example, leaning on or grabbing objects), and 25 points indicating the patient was able to complete movement normally. The total score was 100 points, with higher scores indicating better trunk control.

The self-care agency of patients in both groups was evaluated 6 months after discharge based on the Exercise of Self-care Agency Scale (ESCA) [14] with items including self-concept, self-care skills, self-care, self-responsibility, and health knowledge level. The total score was 270 points, with higher scores indicating better self-care agencies.

The quality of life before and after the intervention of both groups was evaluated by the Generic Quality of Life Inventory-74 (GQOL-74) [15], which included 15 items. The total score was 100 points, and higher scores representing a higher quality of life.

Various three-dimensional gait parameters before and after the intervention of patients were evaluated by the GaitviewAFA-50 gait analyzer (made by Hongtaisheng Health Technology Co., Ltd.), which included pace, gait period, and support phase.

### 2.9. Statistical Methods

The statistical analysis and processing of experimental data was conducted by SPSS21.0 software. The picture drawing of data was completed by GraphPad Prism 7 (GraphPad Software, San Diego, USA). Categorical data were expressed as (*n* (%)) and compared by the *X*^2^ test. Continuous data were expressed as the ($\bar{x}$ ± *s*) and compared by the Student's *t*-tests. Differences were considered statistically significant at *P* < 0.05.

## 3. Results

### 3.1. Comparison of FMA Scores and MBI Scores before and after Intervention between the Two Groups

After intervention, the FMA scores and MBI scores of patients in group A were significantly higher than those in group B (*P* < 0.05) (Table 2).

### 3.2. Comparison of ADL Scores at Different Times between the Two Groups

The ADL scores at T1, T2, and T3 of group A were significantly higher than those of group B (*P* < 0.05) (Figure 1).

### 3.3. Comparison of TCT Scores at Different Times between the Two Groups

The TCT scores at T1, T2, and T3 of group A were significantly higher than those of group B (*P* < 0.05)(Figure 2).

### 3.4. Comparison of ESCA Scores at 6 Months after Discharge between the Two Groups

The self-concept, self-care skills, self-care, self-responsibility, health knowledge level, and total scores at 6 months after discharge of patients in group A were significantly higher than those in group B (*P* < 0.05) (Table 3).

### 3.5. Comparison of GQOL-74 Scores before and after Intervention between the Two Groups

The GQOL-74 scores after intervention of both groups were significantly higher than those before intervention (*P* < 0.05), and those of group A were significantly higher than those of group B (*P* < 0.05) (Figure 3).

### 3.6. Comparison of Various Three-Dimensional Gait Parameters before and after Intervention between the Two Groups

After intervention, patients in group A presented significantly higher walking speed and gait period and lower support phase when compared with group B (*P* < 0.05) (Table 4).

## 4. Discussion

An acute stroke is a kind of acute cerebrovascular circulation disorder that results from various causes. According to the latest WTO data [16], the prevalence of acute strokes around the world is increasing year by year, with an annual growth rate of about 90,000. Although the mortality of patients has been reduced to a certain extent due to the continuous progress of treating cardiovascular and cerebrovascular diseases, most of the survivors still have different dysfunctions left behind, especially dyskinesia. The incidence of upper limb dyskinesia in acute stroke patients is 53–76%, of which about 85% of these patients cannot fully recover after 6 months of stroke, and about 60% of them cannot achieve free movement. The upper limb requires more precise movement and has a cerebral cortex area twice as large as that of the lower limb. As a result, the recovery of the upper limb motor function is slower, which reduces the ability to do daily life as well as the enthusiasm for training to a certain extent and prolongs the rehabilitation process of the patients. Therefore, the rehabilitation of upper limb motor function has become the key of healing treatment for acute stroke patients [17–19].

In the process of limb movement of acute stroke patients, the brain nerve first transmits the motor signal, and then the muscle innervates the nerve reflex contraction for movement. So the concept of rehabilitation treatment for stroke patients with limb motor dysfunction is to reconstruct the normal movement mode from the brain to the muscle group [20–22]. A large number of studies have shown that CIMT can effectively improve the limb motor function of brain stroke patients, and with the help of medical imaging diagnosis, people have found that it can also reconstitute the motor function area of the cerebral cortex.

The results of the study showed that patients in group A given the combined nursing care intervention obtained significantly better ADL scores, TCT scores, and GQOL-74 scores than before, and their waking speed, gait period, and support phase were significantly better than those of patients in group B, indicating that the combined nursing care mode could obviously improve the ADL for acute stroke patients, promote trunk control and body coordination, and ensure a better quality of life. Also, the ESCA scores of patients in group A were significantly higher than those in group B, meaning that patients mastered more knowledge about the administration and nursing of acute stroke, understood the disease more correctly, and improved their self-care ability with the help of continuous care. In this study, continuous care combined with CIMT under a COM-B health platform was performed to stroke patients in group A, who obtained significantly higher FMA scores and MBI scores than those in group B (*P* < 0.001), showing that the combined intervening measure could improve the rehabilitation of upper limb motor function for stroke patients. It was speculated that the continuous nursing mode could better implement the rehabilitation measures by strengthening the nursing management of stroke patients in the rehabilitation period and urging the patients to carry out rehabilitation treatment every day, and with the help of CIMT, patients' cortical activity was triggered and enhanced by repeated training, thus stimulating the hemiplegia limbs and promoting the excitability and reactivity of the nerve system of the affected side, as well as improving the hemiplegia limb movement. APARICIO and others [23] pointed out in the literature that “after performing CIMT combined with acupuncture in stages to patients with paralytic limbs after intracranial aneurysm surgery, the MBI was 75.43 ± 5.34, which was significantly higher than those given conventional rehabilitation treatment (68.37 ± 5.41),” indicating that CIMT could largely promote the recovery of limb function for hemiplegic patients.

In conclusion, continuous care combined with CIMT under a health platform can obviously improve the limb motor function and the quality of life for acute stroke patients, which is worthy of application and promotion.

## Figures and Tables

**Figure 1:** Comparison of ADL scores at different times between the two groups ($\bar{x}$ ± *s*). Note: the horizontal axis indicates T0, T1, T2, and T3, and the vertical axis indicates the ADL score (points); the ADL scores at T0, T1, T2, and T3 of patients in group A were (31.47 ± 5.64), (44.52 ± 4.87), (53.47 ± 4.63), and (62.59 ± 4.78), respectively; the ADL scores at T0, T1, T2, and T3 of patients in group B were (31.56 ± 5.58), (37.19 ± 4.54), (46.32 ± 4.86), and (55.32 ± 4.61), respectively; ^*∗*^indicates that the difference in ADL scores at T1 between the two groups was significant (*t* = 6.420，*P* < 0.001); ^*∗∗*^indicates that the difference in ADL scores at T2 between the two groups was significant (*t* = 6.211, *P* < 0.001); and ^*∗∗∗*^indicates that the difference in ADL scores at T3 between the two groups was significant (*t* = 6.383，*P* < 0.001).

**Figure 2:** Comparison of TCT scores at different times between the two groups ($\bar{x}$±*s*). Note: the horizontal axis indicates T0, T1, T2, and T3, and the vertical axis indicates the TCT score (points); the TCT scores at T0, T1, T2, and T3 of patients in group A were (46.32 ± 5.17), (58.36 ± 5.63), (74.77 ± 5.46), and (84.32 ± 5.12), respectively; the TCT scores at T0, T1, T2, and T3 of patients in group B were (46.35 ± 5.21), (53.86 ± 5.57), (63.86 ± 5.26), and (75.47 ± 4.93), respectively; ^*∗*^indicates that the difference in TCT scores at T1 between the two groups was significant (*t* = 3.313, *P* = 0.002); ^*∗∗*^indicates that the difference in TCT scores at T2 between the two groups was significant (*t* = 8.391, *P* < 0.001); and ^*∗∗∗*^indicates that the difference in TCT scores at T3 between the two groups was significant (*t* = 7.260, *P* < 0.001).

**Figure 3:** Comparison of GQOL-74 scores before and after intervention between the two groups ($\bar{x}$±*s*, points). Note: the horizontal axis indicates before and after intervention, and the vertical axis indicates the GQOL-74 score (points); the GQOL-74 scores before and after intervention of patients in group A were (46.33 ± 5.78) and (72.13 ± 4.69), respectively; the GQOL-74 scores before and after intervention of patients in group B were (46.37 ± 5.75) and (63.19 ± 4.72), respectively; ^*∗*^indicates that the GQOL-74 scores before and after intervention of patients in group A were significantly different (*t* = 20.211, *P* < 0.001); ^*∗∗*^indicates that the GQOL-74 scores before and after intervention of patients in group B were significantly different (*t* = 13.184, *P* < 0.001); and ^*∗∗∗*^indicates that the GQOL-74 scores after intervention of both groups were significantly different (*t* = 7.834, *P* < 0.001).

**Table 1:** Comparison of patients' clinical characteristics between the two groups (*n* (%), ($\bar{x}$ ± *s*)).

Category	Group A (*n* = 34)	Group B (*n* = 34)	*χ* ^2^/t	*P*
Gender			0.059	0.808
Male	19 (55.88%)	18 (52.94%)		
Female	15 (44.12%)	16 (47.06%)		
Mean age (years)	53.46 ± 3.26	53.52 ± 3.28	0.076	0.940
Mean course of disease (months)	4.53 ± 1.46	4.48 ± 1.49	0.140	0.889
Hemiplegic side of upper limbs			0.258	0.612
Left	11 (32.35%)	13 (38.24%)		
Right	23 (67.65%)	21 (61.76%)		
Stroke type			0.059	0.808
Cerebral hemorrhage	15 (44.12%)	16 (47.06%)		
Cerebral infarction	19 (55.88%)	18 (52.94%)		
Residence			1.472	0.225
Cities and towns	19 (55.88%)	14 (41.18%)		
Villages	15 (44.12%)	20 (58.82%)		

**Table 2:** Comparison of FMA scores and MBI scores before and after intervention between the two groups ($\bar{x}$ ± *s*).

Group	*n*	FMA score (points)		MBI score (points)	
		Before	After	Before	After
Group A	34	23.47 ± 8.62	38.42 ± 7.62	62.16 ± 8.72	78.63 ± 6.52
Group B	34	23.52 ± 8.57	31.22 ± 7.25	62.21 ± 8.75	70.24 ± 6.48
*t*		0.024	3.992	0.024	5.322
*P*		0.981	<0.001	0.981	<0.001

**Table 3:** Comparison of ESCA scores at 6 months after discharge between the two groups ($\bar{x}$±*s*, points).

Group	*n*	Self-concept	Self-care skills	Self-care	Self-responsibility	Health knowledge level	Total score
Group A	34	24.25 ± 3.18	25.26 ± 3.18	123.17 ± 6.82	26.31 ± 3.18	48.86 ± 2.35	247.85 ± 18.71
Group B	34	18.22 ± 2.17	20.31 ± 3.15	102.43 ± 6.37	17.53 ± 3.26	41.62 ± 2.41	200.11 ± 17.36
*t*		9.133	6.448	12.959	11.242	12.541	10.907
*P*		<0.001	<0.001	<0.001	<0.001	<0.001	<0.001

**Table 4:** Comparison of various three-dimensional gait parameters before and after intervention between the two groups ($\bar{x}$±*s*).

Group	*n*	Walking speed (cm/s)		Gait period (s)		Support phase (%)	
		Before	After	Before	After	Before	After
Group A	34	13.26 ± 3.27	52.31 ± 4.36	1.24 ± 0.17	1.64 ± 0.22	81.24 ± 8.73	64.52 ± 5.37
Group B	34	13.31 ± 3.25	45.72 ± 4.27	1.26 ± 0.19	1.43 ± 0.24	81.28 ± 8.76	72.15 ± 5.26
*t*		0.063	6.297	0.457	3.761	0.019	5.918
*P*		0.950	<0.001	0.649	<0.001	0.985	<0.001

## Data Availability

Data to support the findings of this study are available on reasonable request from the corresponding author.
